The article "Estimate Stress-Strength Reliability Model Using Rayleigh and Half-Normal Distribution" was published in 2021. Journal: Comput Intell Neurosci.

# Estimate Stress-Strength Reliability Model Using Rayleigh and Half-Normal Distribution

**DOI:** 10.1155/2021/7653581

**Published:** 2021-07-05

**Authors:** Osama Abdulaziz Alamri, M. M. Abd El-Raouf, Eman Ahmed Ismail, Zahra Almaspoor, Basim S. O. Alsaedi, Saima Khan Khosa, M. Yusuf

**Affiliations:** ^1^Department of Statistics, Faculty of Science, University of Tabuk, Tabuk 71491, Saudi Arabia; ^2^Basic and Applied Science Institute, Arab Academy for Science, Technology and Maritime Transport (AASTMT), Alexandia, Egypt; ^3^College of International Transport and Logistics, Arab Academy for Science, Technology and Maritime Transport, Smart Village Campus, Cairo, Egypt; ^4^Department of Statistics, Yazd University, P.O. Box 89175-741, Yazd, Iran; ^5^Department of Statistics, Bahauddin Zakariya University, Multan, Pakistan; ^6^Department of Mathematics, Faculty of science, Helwan University, Cairo, Egypt

## Abstract

In the field of life testing, it is very important to study the reliability of any component under testing. One of the most important subjects is the “stress-strength reliability” term which always refers to the quantity *P* (*X* > *Y*) in any statistical literature. It resamples a system with random strength (*X*) that is subjected to a random strength (*Y*) such that a system fails in case the stress exceeds the strength. In this study, we consider stress-strength reliability where the strength (*X*) follows Rayleigh-half-normal distribution and stress (*Y*_1_, *Y*_2_, *Y*_3_, and *Y*_4_) follows Rayleigh-half-normal distribution, exponential distribution, Rayleigh distribution, and half-normal distribution, respectively. This effort comprises determining the general formulations of the reliabilities of a system. Also, the maximum likelihood estimation approach and method of moment (MOM) will be utilized to estimate the parameters. Finally, reliability has been attained utilizing various values of stress and strength parameters.

## 1. Introduction

The life of a component is described using the stress-strength models, in reliability theory, that is including a random strength (*X*) which is subjected to a random stress (*Y*). The failure of a component is occurred instantaneously when the stress level applied to it exceeds the level of the strength. Thus, the component reliability is measured by *R*=*P*(*Y* < *X*). This measurement has a variety of applications, most notably in the engineering industry, such as the degradation of rocket motors and structures, the fatigue failure of aircraft structures, the ageing of concrete pressure vessels, and static fatigue of ceramic components. Therefore, the estimation of *R*=*P*(*Y* < *X*) has a great importance in the practical applications. The literature demonstrates that reliability estimation (*R*) has already been performed when the distributions of (*X*) and (*Y*) are Weibull, exponential, or log normal.

Church and Harris [1] firstly introduced the term stress-strength. Many authors have adopted various distributions types for stress and strength. The works of Church and Harris, Surles and Padgett [2], Raqab and Kundu [3], Mokhlis [4], and Saraçoğlu et al. [5] contain the discussion of the estimation problems of the stress-strength reliability model for different distributions. Recently, a review of all methods and results on the stress-strength reliability have presented by Kotz et al. [6]. Bayes estimators and reliability function and the parameters of the Consul, Geeta, and size-biased Geeta distributions are obtained by Khan Adil and Jan [7]. Akman et al. [8] studied the estimation of reliability using a finite mixture of inverse Gaussian distributions. The estimation of *R*=*P*(*Y* < *X*) is studied by AI-Hussaini [9] based on a finite mixture of lognormal components. For more reading, see [10–14].

## 2. Finite Mixture of Rayleigh and Half-Normal Distribution

The Rayleigh-half-normal distribution is denoted as **RHN**(*θ*) by Abd El-Monsef and Abd El-Raouf [15]. A mixture of Rayleigh and half-normal distribution with a parameter $\left(1/\sqrt{2\theta }\right)$ is used to represent this model:

(1) $$\begin{array}{c} f\left(x,\;\theta \right)=Kf_{R}\left(\frac{x\cdot 1}{\sqrt{2\theta }}\right)+\left(1-K\right)f_{\text{HN}}\;\left(\frac{x\cdot 1}{\sqrt{2\theta }}\right)\\ =K\left(2\theta xe^{-\theta x^{2}}\right)+\left(1-K\right)\left(2\;\sqrt{\frac{\theta }{\pi }}\;e^{-\theta x^{2}}\right), \end{array}$$

where $K=\left(1/\left(1+\sqrt{\pi \theta }\right)\right)$.

Thus, the Rayleigh-half normal distribution probability density function (pdf) is given by

(2) $$\begin{array}{c} f\left(x,\;\theta \right)=\frac{2\theta \left(x+1\right)e^{-\theta x^{2}}}{1+\sqrt{\pi \theta }},\;x,\theta >0. \end{array}$$

The corresponding cumulative distribution function is given by

(3) $$\begin{array}{c} F\left(x,\;\theta \right)=\frac{1-e^{-\theta x^{2}}+\sqrt{\pi \theta }\text{erf}\left(\sqrt{\theta }x\right)}{1+\sqrt{\pi \theta }},\;x,\theta >0, \end{array}$$

where erf(*u*) is the Gauss error function defined as

(4) $$\begin{array}{c} \text{erf}\left(u\right)=\frac{2}{\sqrt{\pi }}\int_{0}^{u}e^{-t^{2}}\text{d}t. \end{array}$$

### 2.1. The Survival Function and the Hazard Function

The reliability function or the survival function *S*(*x*) tests the chance of occurring of a breakdown of units beyond certain given point in time. For monitoring, a unit lifetime across the support of its lifetime distribution; generally, the probability that an item will work properly for a specified time period with no failure is the survival function. The definition of the survival function is represented as follows:

(5) $$\begin{array}{c} S\left(x\right)=1-F\left(x\right)=\frac{e^{-\theta x^{2}}+\sqrt{\pi \theta }\text{erfc}\left(\sqrt{\theta }x\right)}{1+\sqrt{\pi \theta }}, \end{array}$$

where erfc(*u*) is the complementary error function, and its definition is

(6) $$\begin{array}{c} \text{erfc}\left(u\right)=1-\text{erf}\left(u\right)=\frac{2}{\sqrt{\pi }}\int_{u}^{\infty }e^{-t^{2}}\text{d}t. \end{array}$$

The definition of the hazard rate function is the ratio between the density function and its survival function, which measures the tendency to die or to fail depending on the reached age, and therefore, it has a critical role in the classification of the distributions of lifetime, so the hazard rate function of the RHN distribution is given by

(7) $$\begin{array}{c} h\left(x\right)=\frac{f\left(x\right)}{S\left(x\right)}=\frac{2\theta \left(1+x\right)}{1+e^{\theta x^{2}}\sqrt{\pi \theta }\text{erf}\left(\sqrt{\theta }x\right)}. \end{array}$$

## 3. Stress-Strength Reliability Computations

In this section, the reliability *R*=*P*(*Y* < *X*) was derived, where the random variables (*X*) and (*Y*) are the independent random variables, where the strength *X* follows Rayleigh-half normal distribution and the stress (*Y*) takes different cases (Rayleigh-half normal distribution, exponential distribution, Rayleigh distribution, and half-normal distribution).

Let (*X*) and (*Y*) be two independent random variables, where (*X*) represents “strength” and (*Y*) represents “stress” and (*X*), and (*Y*) follows a joint pdf *f*(*x*, *θ*); thus, the component reliability is

(8) $$\begin{array}{c} R=P\left(Y<X\right)=\int_{-\infty }^{\infty }\int_{-\infty }^{x}f\left(x,y\right)\text{d}y\text{d}x. \end{array}$$

In case that the random variables are statistically independent, then *f*(*x*, *y*)=*f*(*x*)*g*(*y*) so that

(9) $$\begin{array}{c} R=\int_{-\infty }^{\infty }\int_{-\infty }^{x}f\left(x\right)g\left(x\right)\text{d}y\text{d}x, \end{array}$$

where *f*(*x*) and *g*(*y*) are pdf's of *X* and *Y*, respectively.

### 3.1. The Stress and the Strength Follows Rayleigh-Half-Normal Distribution

As the strength *X* ~ RHN(*θ*) and *Y*_1_ ~ RHN(*θ*_1_), they are independent random variables with pdf *f* (*x*) and *g*(*y*_1_), respectively:

(10) $$\begin{array}{c} f\left(x\right)=\frac{2\theta \left(x+1\right)e^{-\theta x^{2}}}{1+\sqrt{\pi \theta }},\;0<\theta \cdot x,\\ g\left(y_{1}\right)=\frac{2\theta_{1}\left(y_{1}+1\right)e^{-\theta_{1}y_{1}^{2}}}{1+\sqrt{\pi \theta_{1}}},\;0<\theta_{1}\cdot y_{1}. \end{array}$$

We derive the reliability *R*=*P*(*Y* < *X*) as follows:

(11) $$\begin{array}{c} R_{1}=P\left(Y<X\right)=\int_{0}^{\infty }\int_{0}^{x}f\left(x\right)g\left(y_{1}\right)\text{d}y\text{d}x\\ =\int_{0}^{\infty }\int_{0}^{x}\left(\frac{2\theta_{1}\left(y_{1}+1\right)e^{-\theta_{1}y_{1}^{2}}}{1+\sqrt{\pi \theta_{1}}}\right)\left(\frac{2\theta \left(x+1\right)e^{-\theta x^{2}}}{1+\sqrt{\pi \theta }}\right)\text{d}y\text{d}x. \end{array}$$

And, we get after the simplification:

(12) $$\begin{array}{c} R_{1}=\frac{\left(1+\sqrt{\pi \theta_{1}}+2\sqrt{\theta \theta_{1}}{\text{Tan}}^{-1}\left(\sqrt{\theta /\theta_{1}}\right)+\left(\sqrt{\pi }\left(\theta -\theta_{1}\right)/\sqrt{\theta +\theta_{1}}\right)-\left(\theta_{1}/\left(\theta +\theta_{1}\right)\right)\right)}{1+\sqrt{\pi \theta }+\sqrt{\pi \theta_{1}}+\pi \sqrt{\theta \theta_{1}}}. \end{array}$$

### 3.2. The Strength Follows RHN Distribution and the Stress Follows Exponential Distribution

In this case, the probability density function (pdf) for the stress *Y*_2_ that follows the exponential distribution is given by

(13) $$\begin{array}{c} g\left(y_{2}\right)=\theta_{2}e^{-y_{1}\theta_{2}},\;y_{2},\theta_{2}>0. \end{array}$$

Then, reliability function *R*_2_ for the independent random variables *X* and *Y*_2_:

(14) $$\begin{array}{c} R_{2}=\int_{0}^{\infty }\int_{0}^{x}\theta_{2}e^{-y_{2}\theta_{2}}\left(\frac{2\theta \left(x+1\right)e^{-\theta x^{2}}}{1+\sqrt{\pi \theta }}\right)\text{d}y\text{d}x,\\ R_{2}=\frac{\sqrt{\pi }}{2\left(\sqrt{\theta }+\sqrt{\pi }\theta \right)}\left(2\theta -\left(2\theta -\theta_{2}\right)e^{\left(\theta_{2}^{2}/4\theta \right)}\text{erfc}\left(\frac{\theta_{2}}{2\sqrt{\theta }}\right)\right), \end{array}$$

where the strength follows RHN distribution.

### 3.3. The Strength Follows RHN Distribution and the Stress Follows Rayleigh Distribution

In this case, the probability density function (pdf) for the stress *Y*_3_ that follows the Rayleigh distribution is given by

(15) $$\begin{array}{c} g\left(y_{3}\right)=\frac{y_{3}}{\theta_{2}^{2}}e^{-\left(y_{3}^{2}/2\theta_{3}^{2}\right)},\;y,\theta_{3}>0. \end{array}$$

Then, reliability function *R*_3_ for the independent random variables *X* and *Y*_3_ is

(16) $$\begin{array}{c} R_{3}=\int_{0}^{\infty }\int_{0}^{x}\left(\frac{y_{3}}{\theta_{3}^{2}}e^{-\left(y_{3}^{2}/2\theta_{3}^{2}\right)}\right)\left(\frac{2\theta \left(x+1\right)e^{-\theta x^{2}}}{1+\sqrt{\pi \theta }}\right)\text{d}y\text{d}x\\ =\frac{2\theta }{\left(1+\sqrt{\pi \theta }\right)}\int_{0}^{\infty }\left(x+1\right)e^{-\theta x^{2}}\left(1-e^{-\left(x^{2}/2\theta_{3}^{2}\right)}\right)\text{d}x,\\ R_{3}=\frac{\theta }{1+\sqrt{\pi \theta }}\;\left(\frac{1}{\theta }+\frac{\sqrt{\pi }}{\sqrt{\theta }}-\frac{2}{2\theta +\left(1/\theta_{3}^{2}\right)}-\frac{\sqrt{2\pi }}{\sqrt{2\theta +\left(1/\theta_{3}^{2}\right)}}\right), \end{array}$$

where the strength follows RHN distribution.

### 3.4. The Strength Follows RHN Distribution and the Stress Follows Half-Normal Distribution

In this case, the probability density function (pdf) for the stress *Y*_4_ that follows half-normal distribution is given by

(17) $$\begin{array}{c} g\left(y_{4}\right)=\left(\frac{\sqrt{2}}{\theta_{4}\sqrt{\pi }}\right)e^{-\left(y_{4}^{2}/2\theta_{4}^{2}\right)},\;y,\theta_{4}>0. \end{array}$$

Then, reliability function *R*_4_ for the independent random variables *X* and *Y*_4_

(18) $$\begin{array}{c} R_{4}=\int_{0}^{\infty }\int_{0}^{x}\left(\left(\frac{\sqrt{2}}{\theta_{4}\sqrt{\pi }}\right)e^{-\frac{y_{4}^{2}}{2\theta_{4}^{2}}}\right)\left(\frac{2\theta \left(x+1\right)e^{-\theta x^{2}}}{1+\sqrt{\pi \theta }}\right)\text{d}y\text{d}x\\ =\frac{2\theta }{\left(1+\sqrt{\pi \theta }\right)}\int_{0}^{\infty }\text{Erf}\left(\frac{x}{\sqrt{2}\theta_{4}}\right)\left(x+1\right)e^{-\theta x^{2}}\text{d}x,\\ R_{4}=\frac{1}{\sqrt{\theta }\left(1+\sqrt{\pi \theta }\right)}\left(\frac{2\theta {\text{Cot}}^{-1}\left(\theta_{4}\sqrt{2\theta }\right)}{\sqrt{\pi }}+\frac{1}{\theta_{4}\sqrt{2+\left(1/\theta \theta_{4}^{2}\right)}}\right), \end{array}$$

where the strength follows RHN distribution.

## 4. Estimation of Stress-Strength Reliability

In the literature, a discussion of the estimation *R* = *P*(*Y* < *X*) when random variables (*X*) and (*Y*) are following the specified distributions have been presented including engineering statistics, quality control, medicine, reliability, biostatistics, and psychology. This quantity for a limited number of cases could be calculated in a closed form (Nadarajah [16] and Barreto-Souza et al. [17]). Several authors including Milan and Vesna [18] have considered the estimation of (*R*) for independent variables and normally distributed (*X*) and (*Y*). Later, a list of papers related to the estimation problem of (*R*) were reported by Greco and Venture [19] when (*X*) and (*Y*) are independent and follow a class of lifetime distributions containing Gamma distributions, exponential, generalized exponential, bivariate exponential, Weibull distribution, Burr type t model, and others.

### 4.1. Method of Moment (MOM) Estimation of *R*

The estimation of reliability is very common in the statistical literature. Now, to compute $\hat{R}$, we need to estimate the parameters *θ* and *θ*_*i*_,  *i*=1,2,3,4, in four cases of stress.

Since the strengths *X* follow RHN (*θ*),the stress have four cases:

- *Y*_1_ follows Rayleigh-half normal distribution with parameter *θ*_1_
- *Y*_2_ follows exponential distribution with parameter *θ*_2_
- *Y*_3_ follows Rayleigh distribution with parameter *θ*_3_
- *Y*_4_ follows half-normal distribution with parameter *θ*_4_; then, their population means are given by

(19) $$\begin{array}{c} \bar{x}=\frac{2\sqrt{\theta }+\sqrt{\pi }}{2\sqrt{\theta }\left(1+\sqrt{\theta \pi }\right)},\\ {\bar{y}}_{1}=\frac{2\sqrt{\theta_{1}}+\sqrt{\pi }}{2\sqrt{\theta_{1}}\left(1+\sqrt{\theta_{1}\pi }\right)},\\ {\bar{y}}_{2}=\frac{1}{\theta_{2}},\\ {\bar{y}}_{3}=\theta_{3}\sqrt{\frac{\pi }{2}},\\ {\bar{y}}_{4}=\theta_{4}\sqrt{\frac{2}{\pi }}. \end{array}$$

The ME's of *θ*, *θ*_1_, *θ*_2_, *θ*_3_,  and *θ*_4_, denoted by $\hat{\theta },{\hat{\theta }}_{1},{\hat{\theta }}_{2},{\hat{\theta }}_{3}$, and ${\hat{\theta }}_{4}$, respectively, can be obtained by solving ($\bar{x}$, ${\bar{y}}_{1}$, ${\bar{y}}_{2}$, ${\bar{y}}_{3}$, and ${\bar{y}}_{4}$) numerically:

(20) $$\begin{array}{c} \hat{\theta }=\frac{{\left(\sum_{i=1}^{m}x_{i}-n\right)}^{2}+n\pi \sum_{i=1}^{m}x_{i}}{2\pi {\left(\sum_{i=1}^{m}x_{i}\right)}^{2}}+\frac{\sqrt{{\left(\sum_{i=1}^{m}x_{i}-n\right)}^{4}+2n\pi \sum_{i=1}^{m}x_{i}{\left(\sum_{i=1}^{m}x_{i}-n\right)}^{2}}}{2\pi {\left(\sum_{i=1}^{m}x_{i}\right)}^{2}},\\ {\hat{\theta }}_{1}=\frac{{\left(\sum_{j=1}^{m}y_{1_{j}}-m\right)}^{2}+m\pi \sum_{j=1}^{m}y_{1_{j}}}{2\pi {\left(\sum_{j=1}^{m}y_{1_{j}}\right)}^{2}}+\frac{\sqrt{{\left(\sum_{j=1}^{m}y_{1_{j}}-n\right)}^{4}+2m\pi \sum_{j=1}^{m}y_{1_{j}}{\left(\sum_{j=1}^{m}y_{1_{j}}-m\right)}^{2}}}{2\pi {\left(\sum_{j=1}^{m}y_{1_{j}}\right)}^{2}},\\ {\hat{\theta }}_{2}=\frac{m}{\sum_{j=1}^{m}y_{2j}},\\ {\hat{\theta }}_{3}=\sqrt{\frac{2}{\pi }}\left(\frac{\sum_{j=1}^{m}y_{3j}}{m}\right),\\ {\hat{\theta }}_{4}=\sqrt{\frac{\pi }{2}}\left(\frac{\sum_{j=1}^{m}y_{4j}}{m}\right). \end{array}$$

The ME of *R*, denoted by ${\hat{R}}_{1}\cdot {\hat{R}}_{2}\cdot {\hat{R}}_{3}$ and ${\hat{R}}_{4}$ is obtained by substitute $\hat{\theta }$ with ${\hat{\theta }}_{1}\cdot {\hat{\theta }}_{2}\cdot {\hat{\theta }}_{3}$ and ${\hat{\theta }}_{4}$ in *R*_1_ · *R*_2_ · *R*_3_ and *R*_4_.

### 4.2. The Maximum Likelihood Estimators of *R*

The maximum likelihood estimator (MLE) is the most popular method for reliability estimation *R*=*p*(*Y* < *X*) because of its generality and flexibility. This method can be used if the joint distribution of the strength (*X*) and the stress (*Y*) is a known function with some unknown parameters.

Suppose *x*_1_ · *x*_2_ · ⋯·*x*_*n*_ is a random sample from RHN distribution with *θ* and *y*_11_ · *y*_12_ · ⋯·*y*_1*m*_ is a random sample from RHN distribution with *θ*_1_. Then, the likelihood function is given by

(21) $$\begin{array}{c} L\left(\theta \cdot \theta_{1};x\cdot y_{1}\right)=2^{n+m}\theta^{n}\theta_{1}^{m}-{\left(1+\sqrt{\pi \theta }\right)}^{n}-{\left(1+\sqrt{\pi \theta_{1}}\right)}^{m}\prod_{i=1}^{n}\left(x_{i}+1\right)e^{-\theta x_{i}^{2}}\prod_{j=1}^{m}\left(y_{1j}+1\right)e^{-\theta_{1}y_{1j}^{2}}. \end{array}$$

And, the log-likelihood function of the observed samples is

(22) $$\begin{array}{c} \ln\;L\left(\theta \cdot \theta_{1}\right)=\left(m+n\right)\ln\left(2\right)+n\;\ln\left(\theta \right)+m\;\ln\left(\theta_{1}\right)-n\;\ln\left(1+\sqrt{\pi \theta }\right)-m\;\ln\left(1+\sqrt{\pi \theta_{1}}\right)-\theta \sum_{i=1}^{n}x_{i}^{2}-\theta_{1}\sum_{j=1}^{m}y_{1j}^{2}+\sum_{i=1}^{n}\ln\left(x_{i}+1\right)+\sum_{j=1}^{m}\ln\left(y_{1j}+1\right). \end{array}$$

By solving the following equations, the MLE of *θ* and *θ*_2_ can be obtained:

(23) $$\begin{array}{c} \frac{\left(\partial \;\ln L\left(\theta \cdot \theta_{1}\right)\right)}{\partial \theta }=\frac{n}{\theta }-\frac{\left(n\sqrt{\pi }\right)}{\left(2\sqrt{\theta }\left(1+\sqrt{\pi \theta }\right)\right)}-\overset{n}{\underset{\left(i=1\right)}{\sum }}x_{i}^{2}=0,\\ \frac{\partial \;\ln L\left(\theta \cdot \theta_{1}\right)}{\partial \theta_{1}}=\frac{m}{\theta_{1}}-\frac{m\sqrt{\pi }}{2\sqrt{\theta_{1}}\left(1+\sqrt{\pi \theta_{1}}\right)}-\sum_{j=1}^{m}y_{1j}^{2}=0. \end{array}$$

The MLEs of *θ* and *θ*_1_ can be obtained, respectively, as

(24) $$\begin{array}{c} \hat{\theta }=\frac{1}{6\pi A^{2}}\left(B+2A\left(A+n\pi \right)+\frac{A^{2}\left(n^{2}\pi^{2}+4A\left(A-4n\pi \right)\right)}{B}\right),\\ {\hat{\theta }}_{1}=\frac{1}{6\pi C^{2}}\left(D+2C\left(C+m\pi \right)+\frac{C^{2}\left(m^{2}\pi^{2}+4C\left(C-4m\pi \right)\right)}{D}\right), \end{array}$$

where *A*=∑_*i*=0_^*n*^*x*_*i*_^2^ ·  *C*=∑_*j*=0_^*m*^*y*_1*j*_^2^,

(25) $$\begin{array}{c} B={\left(8A^{6}-48\pi nA^{5}+51\pi^{2}n^{2}A^{4}-\pi^{3}n^{3}A^{3}+3\sqrt{3}\pi^{3/2}\sqrt{n^{3}A^{7}\left(-16A^{2}+71\pi nA-2\pi^{2}n^{2}\right)}\right)}^{1/3}, \end{array}$$

$D={\left(8C^{6}-48\pi mC^{5}+51\pi^{2}m^{2}C^{4}-\pi^{3}m^{3}C^{3}+3\sqrt{3}\pi^{3/2}\sqrt{m^{3}C^{7}\left(-16C^{2}+71\pi mC-2\pi^{2}m^{2}\right)}\right)}^{1/3}$.

Then, the maximum likelihood estimator of *R* when the strength *X* follows RHN(*θ*) distribution and stress *Y* follows RHN(*θ*_1_) distribution is given as

(26) $$\begin{array}{c} {\hat{R}}_{1}=\frac{\left(1+\sqrt{\pi {\hat{\theta }}_{1}}+2\sqrt{\hat{\theta }{\hat{\theta }}_{1}}{\text{Tan}}^{-1}\left(\sqrt{\left(\hat{\theta }/{\hat{\theta }}_{1}\right)}\right)+\left(\sqrt{\pi }\left(\hat{\theta }-{\hat{\theta }}_{1}\right)/\sqrt{\hat{\theta }+{\hat{\theta }}_{1}}\right)-\left({\hat{\theta }}_{1}/\left(\hat{\theta }+{\hat{\theta }}_{1}\right)\right)\right)}{1+\sqrt{\pi \hat{\theta }}+\sqrt{\pi {\hat{\theta }}_{1}}+\pi \sqrt{\hat{\theta }{\hat{\theta }}_{1}}}. \end{array}$$

Similarly, we perform the same steps to find (MLE) in other cases; we can obtain

(i) When the stress *Y*_2_ that follows the exponential distribution with parameter *θ*_2_, the MLE of *R*_2_ is given as
  (27) $$\begin{array}{c} {\hat{R}}_{2}=\frac{\sqrt{\pi }}{2\left(\sqrt{\hat{\theta }}+\sqrt{\pi }{\hat{\theta }}_{2}\right)}\left(2\hat{\theta }-\left(2\hat{\theta }-{\hat{\theta }}_{2}\right)e^{\left({\hat{\theta }}_{2}^{2}/4\hat{\theta }\right)}\text{Erfc}\left(\frac{{\hat{\theta }}_{2}}{2\sqrt{\hat{\theta }}}\right)\right), \end{array}$$
where the strength *X* follows Rayleigh-half-normal distribution with parameter *θ*.
(ii) When the stress *Y*_3_ that follows Rayleigh distribution with parameter *θ*_3_ and the strength *X* follows Rayleigh-half-normal distribution with parameter *θ*, the MLE of *R*_3_ is given as
  (28) $$\begin{array}{c} {\hat{R}}_{3}=\frac{\hat{\theta }}{1+\sqrt{\pi \hat{\theta }}}\left(\frac{1}{\hat{\theta }}+\frac{\sqrt{\pi }}{\sqrt{\hat{\theta }}}-\frac{2}{2\hat{\theta }+\left(1/{\hat{\theta }}_{3}^{2}\right)}-\frac{\sqrt{2\pi }}{\sqrt{2\hat{\theta }+\left(1/{\hat{\theta }}_{3}^{2}\right)}}\right). \end{array}$$
(iii) When the stress *Y*_4_ that follows half-normal distribution with parameter *θ*_4_, the M. L. E of *R*_2_ is given as

(29) $$\begin{array}{c} {\hat{R}}_{4}=\frac{1}{\sqrt{\hat{\theta }}\left(1+\sqrt{\pi \hat{\theta }}\right)}\;\left(\frac{2\hat{\theta }{\text{Cot}}^{-1}\left({\hat{\theta }}_{2}\sqrt{2\hat{\theta }}\right)}{\sqrt{\pi }}+\frac{1}{{\hat{\theta }}_{4}\sqrt{2+\left(1/\hat{\theta }{\hat{\theta }}_{4}^{2}\right)}}\right), \end{array}$$

where the strength *X* follows Rayleigh-half-normal distribution with parameter *θ*.

## 5. Numerical Evaluation

In different cases, the system reliability *R* has evaluated for some specific values of the parameters involved in the expression of *R*.

### 5.1. Case 1: Strength and Stress Follows RHN Distribution

From Table 1 and Figures 1 and 2, it is noticed that, with the increase in the strength parameter values, the reliability value decreases. If the stress parameter increases, then the value of reliability increases.

### 5.2. Case 2: Strength Follows RHN Distribution and Stress Follows Exponential Distribution

From Table 2 and Figures 3 and 4, it is observed that if the strength parameter increases then the value of reliability increases. If the stress parameter increases, then the value of reliability increases.

### 5.3. Case 3: Strength Follows RHN Distribution and Stress Follows Rayleigh Distribution

From Table 3 and Figures 5 and 6, it is noticed that, with increasing the value of the strength and stress parameter, the reliability value decreases.

### 5.4. Case 4: Strength Follows RHN Distribution and Stress Follows Half-Normal Distribution

From Table 4 and Figures 7 and 8, it is noticed that, with increasing the value of the strength and stress parameter, the reliability value decreases.

### 5.5. Simulation Study

In this section, some results are represented depending on Monte-Carlo simulation, for comparing the estimates of (*R*) performance using MLE and MOM estimators fundamentally for many sample sizes. The following sample sizes are considered; (*n*, *m*) = (5, 5), (10, 10), (20, 20), (30, 30), (40, 40), (50, 50), and (100, 100). From each sample, the estimates are computed for the parameters using MLE and method of moment estimation. Once the parameters are estimated, the estimates of *R*_1_ is obtained. The average biases of *R*_1_ is reported in Table 5 and mean squared errors (MSEs) of *R*_1_ are in Table 6.

The first row includes the average bias of *R*_1_ using the MLE and second row includes the average bias of *R*_1_ using the MOM, in each cell.

The first row includes the average MSE of *R*_1_ using the MLE and second row includes the average MSE of *R*_1_ using the MOM, in each cell.

## 6. Conclusions

The proposed model in this paper, the stress-strength reliability has been studied for Rayleigh-half normal when the strength (*X*) follows Rayleigh-half normal distribution, and the stress (*Y*) takes Rayleigh-half normal distribution, exponential distribution, Rayleigh distribution, and half-normal distribution. Based on the computations and graphs, (i) it has been noticed that when the stress parameter is increased, the reliability value lowers, and when the strength parameter is increased, the reliability value increases. The numerical assessment demonstrates that increasing the stress parameter decreases the dependability value in case (ii), whereas increasing the strength parameter increases the reliability value. In cases (iii) and (vi), increasing the stress parameter decreases the reliability value, whereas increasing the strength parameter increases it. A comparison is carried out between two methods of reliability estimation *R*=*P*(*X* > *Y*) when (*Y*) and (*X*) both follow Rayleigh-half normal distributions for various parameters scale. We provide MLE and MOM procedure for estimating the unknown parameters that are used for reliability estimation (*R*). Based on the simulation findings, we can conclude that MLE outperforms MOM in terms of average bias and average MSE for a variety of parameter choices.

## Figures and Tables

**Figure 1:** Variation in *R*_1_ for constant stress.

**Figure 2:** Variation in *R*_1_ for constant strength.

**Figure 3:** Variation in *R*_2_ for constant stress.

**Figure 4:** Variation in *R*_2_ for constant strength.

**Figure 5:** Variation in *R*_3_ for constant stress.

**Figure 6:** Variation in *R*_3_ for constant strength.

**Figure 7:** Variation in *R*_4_ for constant stress.

**Figure 8:** Variation in *R*_4_ for constant strength.

**Table 1:** Variation in *R*_1_ when strength and stress has RHN distribution.

*θ*	*θ*_1_									
	**0.1**	**0.2**	**0.3**	**0.4**	**0.5**	**0.6**	**0.7**	**0.8**	**0.9**	**1**
**0.1**	0.208	0.359	0.472	0.558	0.624	0.677	0.718	0.752	0.780	0.803
**0.2**	0.149	0.267	0.364	0.442	0.507	0.561	0.606	0.645	0.678	0.706
**0.3**	0.121	0.222	0.307	0.379	0.440	0.493	0.538	0.577	0.611	0.641
**0.4**	0.105	0.194	0.271	0.337	0.395	0.445	0.490	0.529	0.563	0.594
**0.5**	0.093	0.174	0.245	0.307	0.362	0.410	0.453	0.491	0.526	0.556
**0.6**	0.085	0.159	0.225	0.284	0.336	0.382	0.424	0.461	0.495	0.526
**0.7**	0.078	0.148	0.210	0.265	0.315	0.360	0.400	0.437	0.470	0.500
**0.8**	0.073	0.138	0.197	0.250	0.297	0.341	0.380	0.416	0.448	0.478
**0.9**	0.068	0.130	0.186	0.237	0.283	0.325	0.363	0.398	0.430	0.459
**1**	0.065	0.124	0.177	0.226	0.270	0.311	0.348	0.382	0.413	0.443

**Table 2:** Variation in *R*_2_ when strength has RHN distribution and stress has Exponential distribution.

*θ*	*θ*_2_									
	**0.1**	**0.2**	**0.3**	**0.4**	**0.5**	**0.6**	**0.7**	**0.8**	**0.9**	**1**
**0.1**	0.500	0.349	0.274	0.228	0.197	0.175	0.157	0.144	0.133	0.124
**0.2**	0.651	0.500	0.412	0.354	0.312	0.280	0.256	0.236	0.219	0.205
**0.3**	0.726	0.588	0.500	0.438	0.392	0.357	0.328	0.304	0.285	0.268
**0.4**	0.772	0.646	0.562	0.500	0.453	0.415	0.384	0.359	0.337	0.318
**0.5**	0.803	0.688	0.608	0.547	0.500	0.462	0.430	0.403	0.380	0.361
**0.6**	0.825	0.720	0.643	0.585	0.538	0.500	0.468	0.441	0.417	0.396
**0.7**	0.843	0.744	0.672	0.616	0.570	0.532	0.500	0.472	0.448	0.427
**0.8**	0.856	0.764	0.696	0.641	0.597	0.559	0.528	0.500	0.476	0.455
**0.9**	0.867	0.781	0.715	0.663	0.620	0.583	0.552	0.524	0.500	0.479
**1**	0.876	0.795	0.732	0.682	0.639	0.604	0.573	0.545	0.521	0.500

**Table 3:** Variation in *R*_3_ when strength has RHN distribution and stress has Rayleigh distribution.

*θ*	*θ*_3_									
	**0.1**	**0.2**	**0.3**	**0.4**	**0.5**	**0.6**	**0.7**	**0.8**	**0.9**	**1**
**0.1**	0.983	0.963	0.941	0.917	0.891	0.864	0.835	0.806	0.777	0.747
**0.2**	0.970	0.936	0.898	0.858	0.816	0.773	0.730	0.687	0.645	0.604
**0.3**	0.959	0.913	0.863	0.810	0.756	0.702	0.650	0.600	0.552	0.508
**0.4**	0.949	0.892	0.831	0.768	0.706	0.645	0.587	0.533	0.483	0.438
**0.5**	0.940	0.874	0.804	0.732	0.662	0.596	0.535	0.479	0.429	0.385
**0.6**	0.932	0.857	0.778	0.700	0.625	0.555	0.492	0.436	0.386	0.343
**0.7**	0.924	0.841	0.755	0.671	0.591	0.519	0.455	0.399	0.351	0.309
**0.8**	0.917	0.826	0.734	0.644	0.562	0.488	0.424	0.368	0.321	0.281
**0.9**	0.910	0.812	0.714	0.620	0.535	0.460	0.396	0.342	0.296	0.257
**1**	0.903	0.799	0.695	0.598	0.511	0.435	0.372	0.318	0.274	0.238

**Table 4:** Variation in *R*_4_ when strength has RHN distribution and stress has half-normal distribution.

*θ*	*θ*_4_									
	**0.1**	**0.2**	**0.3**	**0.4**	**0.5**	**0.6**	**0.7**	**0.8**	**0.9**	**1**
**0.1**	0.989	0.977	0.964	0.950	0.934	0.918	0.901	0.884	0.866	0.848
**0.2**	0.981	0.960	0.937	0.913	0.888	0.862	0.835	0.808	0.781	0.755
**0.3**	0.974	0.946	0.915	0.883	0.850	0.816	0.783	0.750	0.718	0.687
**0.4**	0.968	0.933	0.896	0.857	0.817	0.778	0.740	0.703	0.668	0.634
**0.5**	0.963	0.921	0.878	0.834	0.789	0.745	0.704	0.664	0.627	0.592
**0.6**	0.957	0.911	0.862	0.812	0.764	0.717	0.672	0.630	0.592	0.557
**0.7**	0.952	0.901	0.847	0.793	0.741	0.691	0.644	0.602	0.562	0.527
**0.8**	0.948	0.891	0.833	0.775	0.720	0.668	0.620	0.576	0.537	0.501
**0.9**	0.943	0.883	0.820	0.759	0.701	0.647	0.598	0.554	0.514	0.479
**1**	0.939	0.874	0.808	0.744	0.683	0.628	0.578	0.533	0.494	0.459

**Table 5:** Average MSE of the simulated estimates of *R*_1_.

(*θ* · *θ*_1_)	(*n*, *m*)						
	(5, 5)	(10, 10)	(20, 20)	(30, 30)	(40, 40)	(50, 50)	(100, 100)
(1, 1)	0.0196	0.0180	−0.0181	−0.0073	−0.0041	−0.0034	0.0005
	−0.0720	−0.0318	−0.0193	0.0138	−0.0084	0.0076	−0.0029

(1, 0.5)	−0.0594	−0.0476	−0.0132	−0.0120	−0.0101	−0.0043	0.0048
	−0.0790	−0.0747	−0.0643	−0.0662	−0.0617	−0.0658	−0.0555

(1, 1.5)	−0.0419	0.0262	0.0172	0.0146	−0.0063	0.0024	0.0011
	0.0678	0.0643	0.0557	0.0478	0.0423	0.0372	0.0370

(1, 2)	−0.0125	0.0115	0.0111	0.0113	−0.0073	0.0044	−0.0015
	0.0800	−0.0777	0.0687	0.0663	0.0656	0.0649	0.0638

(0.5, 1)	0.0252	0.0146	0.0122	−0.0097	−0.0030	−0.0018	0.0011
	0.0743	0.0737	0.0686	0.0656	0.0654	0.0639	0.0627

(1.5, 1)	0.0594	−0.0090	0.0076	−0.0064	0.0062	0.0019	0.0019
	−0.0807	−0.0413	−0.0402	−0.0364	−0.0352	−0.0164	0.0125

(2, 1)	0.0153	0.0066	0.0066	0.0061	0.0048	0.0048	0.0045
	−0.0997	−0.0726	−0.0719	−0.0647	−0.0624	−0.0618	−0.0584

**Table 6:** Average MSE of the simulated estimates of *R*_1_.

(*θ* · *θ*_1_)	(*n*, *m*)						
	(5, 5)	(10, 10)	(20, 20)	(30, 30)	(40, 40)	(50, 50)	(100, 100)
(1, 1)	0.0051	0.0020	0.0020	0.0013	0.0010	0.0005	0.0003
	0.0159	0.0104	0.0090	0.0035	0.0024	0.0020	0.0013

(1, 0.5)	0.0123	0.0095	0.0037	0.0033	0.0025	0.0018	0.0009
	0.0148	0.0112	0.0051	0.0049	0.0046	0.0044	0.0044

(1, 1.5)	0.0077	0.0072	0.0044	0.0030	0.0022	0.0020	−0.0001
	0.0135	0.0091	0.0054	0.0051	0.0034	0.0021	0.0020

(1, 2)	0.0055	0.0050	0.0048	0.0033	0.0022	0.0019	−0.0003
	0.0115	0.0086	0.0059	0.0059	0.0049	0.0049	0.0009

(0.5, 1)	0.0090	0.0038	0.0038	0.0036	0.0031	0.0024	0.0010
	0.0092	0.0087	0.0070	0.0050	0.0050	0.0048	0.0046

(1.5, 1)	0.0147	0.0097	0.0024	0.0024	−0.0018	0.0014	−0.0008
	0.0221	−0.0124	−0.0090	0.0062	0.0027	0.0022	0.0014

(2, 1)	0.0121	0.0064	0.0059	0.0030	0.0024	0.0018	−0.0003
	0.0478	−0.0272	0.0256	−0.0145	−0.0076	0.0050	0.0010

## Data Availability

All data used to support the findings of the study are available within the article.
